The article "Mortality prediction in ICU Using a Stacked Ensemble Model" was published in 2022. Journal: Comput Math Methods Med.

# Mortality prediction in ICU Using a Stacked Ensemble Model

**DOI:** 10.1155/2022/3938492

**Published:** 2022-11-28

**Authors:** Na Ren, Xin Zhao, Xin Zhang

**Affiliations:** School of Mathematics, Southeast University, Nanjing 210096, China

## Abstract

Artificial intelligence (AI) technology has huge scope in developing models to predict the survival rate of critically ill patients in the intensive care unit (ICU). The availability of electronic clinical data has led to the widespread use of various machine learning approaches in this field. Innovative algorithms play a crucial role in boosting the performance of models. This study uses a stacked ensemble model to predict mortality in ICU by incorporating the clinical severity scoring results, in which several machine learning algorithms are employed to compare the performance. The experimental results show that the stacked ensemble model achieves good performance compared with the model without integrating the severity scoring results, which has the area under curve (AUC) of 0.879 and 0.862, respectively. To improve the performance of prediction, two feature subsets are obtained based on different feature selection techniques, labeled as SetS and SetT. Evaluation performances show that the SEM based on the SetS achieves a higher AUC value (0.879 and 0.860). Finally, the SHapley Additive exPlanations (SHAP) analysis is employed to interpret the correlation between the risk features and the outcome.

## 1. Introduction

With the progress of medical technology and the arrival of aging society, the demand for critical care is increasing. The intensive care unit (ICU) is a vital department, in which patients with severe conditions will receive continuous, efficient, and intensive care to improve their health conditions. Generally, a critically ill patient requires special monitoring equipment and the support of multiple medical staff. The cost of patients in ICU is approximately 3.5 times that of patients in regular care [1]. The regular operation of ICU depends on the availability of adequate medical resources [2, 3]. In addition, timely treatment of critical patients often involves many factors, such as the accuracy of disease diagnosis, the efficiency of treatment, and the severity of the disease. However, the growth of medical resource supply and medical investment is relatively limited with the increasing number of patients. From the point of hospital management, the above work mainly focuses on optimal allocation and operational decision assistance with predictive modeling [1]. In recent years, increasing attention has been devoted to the improvement of efficiency in ICU. Fortunately, with the widespread use of electronic health records and the rise of intelligent technology, the effect of prediction has been constantly updated.

The article "Mortality prediction in ICU Using a Stacked Ensemble Model" was published in 2022. Journal: Comput Math Methods Med.

Severity scoring system is a commonly used technique in clinical practice, in which the scores are calculated based on physiological assessment of patients. The Acute Physiology and Chronic Health Evaluation (APACHE) proposed by Knous [4] is a commonly used evaluation system that evaluates critical patients in ICU based on severity scores. It has proven to be an effective tool in measuring the severity among critical patients. APACHE 2 is widely used in ICU but has the problem of overestimating the mortality rate [4, 5]. APACHE 4 system [6] was developed by using the first 24 hours of information, in which the severity score is calculated by summing of the acute physiology score, the age score, and the numerical score. [7] used the APACHE 4 to model the prediction of mortality rate and give a comparison with other scoring results. There are also other conventional evaluation approaches for scoring severity, such as Sequential Organ Failure Assessment (SOFA), Glasgow Coma Scale (GCS), and CT score [7].

Artificial intelligence technology has considerable scope in developing models to predict the survival rate of critically ill patients in the intensive care unit (ICU). The availability of electronic clinical data has led to the widespread use of various machine learning approaches in this field. Fortunately, the development of medical technology and the abundance of electronic records on monitoring indicators provide a reliable and rich source for the development of new mortality prediction methods. Medical Information Mart for Intensive Care 3 (MIMIC-3) is a freely available database that includes healthy data records from over forty thousand patients who stayed in the critical care units of the Beth Israel Deaconess Medical Center (BIDMC) between 2001 and 2012 [8]. The rapid improvement of data mining and machine learning methods has made significant achievements in classification and prediction tasks. Recently, intensive studies have been proposed based on the MIMIC-3 database. [9] proposed an explainable machine learning algorithm for risk factor analysis of in-hospital mortality based on the dataset with 2970 enrolled patients which are selected from the MIMIC-3 database.

The combination of big data technology and clinical severity scoring approaches plays a crucial role in improving the quality of treatment [10, 11]. Accurate analysis of critically ill patients not only helps to improve treatment efficiency and survival rate but also provides relevant information for medical resource allocation and management. Motivated by the existed techniques, a mortality prediction model (SEM) is proposed by combining the clinical severity scoring result with machine learning model using stacked ensemble technique. The hierarchical framework of stacked integration enables the existing severity scoring results to be weighted with the results based on different machine learning models. The detail algorithm procedure is listed in Section 3.

The article "Mortality prediction in ICU Using a Stacked Ensemble Model" was published in 2022. Journal: Comput Math Methods Med.

The contributions of this study include the following:

1. A series of preprocessing procedures executed on the public clinical dataset
2. In terms of feature selection, the subset features (SetS) and the transformed feature set (SetT) are developed
3. Several weak learners (AL) based on APACHE severity scoring results are learned using the machine learning methods
4. A mortality prediction model combined with APACHE severity score results is established by using stack integration technique
5. To interpret the correlation between features and the outcome, the SHAP analysis is employed to give the ranking of the importance features

The rest of this research is organized as follows: materials and methods are given in Section 3. Experiment processes and results are given in Section 4. Conclusions and some extended future work are listed in Section 5. All experiments in our study are performed using R software on a system with i5 Processor (8th generation), RAM of 8 GB, SSD of 256 GB. The detail packages used in the experiments are listed at the first paragraph in Section 4.

## 2. Literature Review

In recent years, data-driven algorithms based on clinical big data have achieved good performance in clinical prediction. Logistic regression (LR) is a well-known linear model that can handle classification tasks. However, the nonlinear structure of the dataset often leads to poor performance in practice [12, 13]. Approaches such as support vector machine (SVM) [11], artificial neural networks (ANN), and Naive Bayes (NB) are widely used in mortality prediction [13]. Recently, tree-based algorithms such as decision tree, random forest (RF), and extreme gradient boosting (XGB) have achieved good classification evaluation in prediction [1, 11, 14]. Deep learning is a complex machine learning algorithm that has achieved remarkable achievements in the field of speech and image recognition. Typical deep learning models include convolutional neural network (CNN), deep belief networks (DBN), and long short term memory network (LSTM [15]. The use of deep learning techniques in healthcare has been limited due to the poor explainability. Recently, [16] introduced a new occlusion-based method to improve the explainability of RNN model in predicting the mortality risk in ICU. In addition to the above methods, it is a good choice to use integration technology to improve the prediction performance of model [12]. Conventional integration techniques mainly include bagging, boosting, and stacking. Random forest is one of the familiar ensemble models, which is based on the bagging ensemble. Different from the other two types of integration models, stacking can aggregate several types of heterogeneous base learners into a metalearner.

The article "Mortality prediction in ICU Using a Stacked Ensemble Model" was published in 2022. Journal: Comput Math Methods Med.

Due to various problems brought by clinical data, mortality prediction often faces significant challenges. To promote the development of clinical big data modeling, various international big data competitions on the theme of mortality prediction were held to boost the development of new algorithms for predicting mortality rate in ICU [17, 18]. The topic of model performance caused by the dataset itself has become an important research topic in the field of information medicine. The main problems faced by common clinical big data are category imbalance, serious missing, and high dimensionality, which usually bring challenges to the improvement of modeling methods and effects. The structure of class imbalance in clinical data often intensively affects the performance of the model [19]. From the data level to the algorithm level, several approaches were proposed to deal with the problem of imbalance. [20] accomplished the detection of rare cases by taking the quantile function of the generalized extreme value distribution as the link function in the framework of XGBoost. [21] proposed a modified cost-sensitive principal component analysis (MCSPCA) method for handling the problem of high-dimension and unbalance existing in the ICU dataset.

Feature selection is critical for developing a model to predict mortality in ICU. The risk of mortality in ICU varies with disease and depends on the monitoring values of different indicators. To determine the critical indicators based on the given monitoring dataset is a crucial factor in determining the prediction performance of the model. Feature selection based on correlation analysis [13] is one of the commonly used methods in research. Based on machine learning algorithms, such as random forest can give the important ranking of features through the corresponding evaluation index. The other conventional approach used to handle feature selection in high dimensionality data is dimensionality reduction, in which the original features are converted to new features using linearly (or nonlinearly) transformation methods. [22] proposed a new interactive feature selection dimension reduction method, and compared it with LASSO, subset selection by validating on the given dataset. [23] developed a novel network-based dimensionality reduction method and applied it to the actual dataset.

The article "Mortality prediction in ICU Using a Stacked Ensemble Model" was published in 2022. Journal: Comput Math Methods Med.

The interpretability of model results plays a key role in future prediction. However, in the field of artificial intelligence, models are often complex or built using an integrated approach, and it is not easy to evaluate the important features that have a significant impact on the results. Explainable AI (XAI) [24] is a burgeoning field that aims to explain how artificial intelligence systems work. The work of AI system could be more reliable and explainable with the progress of XAI techniques. As a commonly used XAI technique, the SHapley Additive exPlanations (SHAP) analysis [25, 26] tries to interpret the prediction of the complex model, in which the variable importance is measured by the mean absolute Shapley value. Variables with positive Shapley values can increase the probability of mortality. The feature importance and partial dependence analysis are obtained using the SHAP evaluator in Section 4. The main characteristics of the related literatures are summarized in Table 1.

In terms of the need for interpretability and the convenience of using computational software, several machine learning models are chosen as base and comparison models in this study. The motivation and focus of this work mainly come from the following points:

1. In addition to promising accuracy, the ML-based model has strong model interpretability
2. Compared to the single technique (such as LR, RF, and XGB), stacked ensemble techniques can improve the prediction performance by weighting the various results
3. Similar to [10], the existing prediction model enriched by incorporating the APACHE score-based result

## 3. Materials and Methods

### 3.1. Data Description

The dataset used in this research is obtained from the 2020 WiDS (Women in Data Science) Challenge [18], which held to establish a model for the prediction of mortality rate in ICU. The data consists of three datasets, training data for 91713 encounters, unlabeled test data for 39308 encounters, and the data table WiDS Datathon 2020 Dictionary. The purpose of this study is to validate the proposed model, so all samples with labels are employed in our study. The data table WiDS Datathon 2020 Dictionary gives supplemental information about the data, including the name of features (e.g., identifier, demographic, and vitals), data types (e.g., numeric and binary), description of each feature, and examples. Feature types consist of identifiers, demographic, vitals, labs, labs blood gas, and APACHE. The type of APACHE has a total of 40 features, including APACHE covariates, APACHE comorbidity, APACHE grouping, and APACHE prediction. The value of features mainly includes continuous type and discrete type.

The article "Mortality prediction in ICU Using a Stacked Ensemble Model" was published in 2022. Journal: Comput Math Methods Med.

Clinical data is often problematic for a variety of reasons. Some feature records are missing due to monitoring device faults. The extent to which patients participate in the monitoring process determines the validity of the monitoring data. In summary, the characteristics of the data are summarized as follows:

1. Class imbalance: the imbalance of class features is a common problem in clinical data. The dataset is severely imbalanced, which includes survival case 83798 compared to the opposite case 7915. Dealing with class imbalance is an essential part of data preprocessing because it leads to poor performance of the model
2. Missing data (MD): the second problem is the high percentage of missing values. The number of cases that have no missing value is 300, which means that the missing problem exists for almost all cases. From the point of feature, the number of complete features is 32, and the value of the missing rate ranges from 0 to 0.92265.  Table 2 gives the examples of feature information and the description of missing percentage. The problem of missing value presents a great challenge for modeling. Handling missing data is an important part of data preprocessing, which determines the performance of the model
3. High dimension: there are 186 features in the original dataset, including 8 category features and 178 numerical features. Critically ill patients in ICU are likely to be monitored simultaneously with multiple monitoring devices for better information. This leads to the redundancy of electronic records. Another problem with high dimensions is the collinearity between features. For example, the value of d1_heart_min indicates the lowest heart rate in the first hour of unit stay, and h1_heart_min indicates the lowest heart rate in the first 24 hours of unit stay, which may have the same trend in the first 24 hours. The problem of high dimension makes modeling complicated and leads to feature interpretation difficult

### 3.2. Data Preprocessing

From different perspectives, the structure of the dataset is complex, which poses challenges for modeling. In order to reduce the impact of various problems, some preprocessing work is needed to improve the quality of the data. It is noted that there are several features which have no contribution to the outcome, such as the features hospital_id, patient_id, and encounter_id. It is found that most continuous features do not have a normal approximation. We choose to delete the outliers based on the concept of quantile. The method used for handling outliers is proposed using the idea of the interquartile range (IQR) [13]. The detailed procedures are given as follows:

(1) $$\begin{array}{c} \text{IQR}=U_{3}-U_{1},\\ \text{Uppe}{\text{r}}_{u}=U_{3}+2*\text{IQR},\\ \text{Lowe}{\text{r}}_{u}=U_{3}-2*\text{IQR},\\ \text{Inpu}{\text{t}}_{u}=\left\{\begin{array}{cc} 1 & \text{Inpu}{\text{t}}_{u}>\text{Uppe}{\text{r}}_{u}\text{orInpu}{\text{t}}_{u}<\text{Uppe}{\text{r}}_{u}\\ 0 & \text{else} \end{array}\right., \end{array}$$

where Input indicates input data, *U*_3_ is the 75% quantile, and *U*_1_ is the 25% quantile. IQR represents the length of a random interval defined by two quantiles. The value is identified as an outlier when the value of the input is equal to 1, and the outliers are replaced by the median of the feature corresponding.

The article "Mortality prediction in ICU Using a Stacked Ensemble Model" was published in 2022. Journal: Comput Math Methods Med.

MD is a common phenomenon in clinical data. The type of MD includes missing at random, missing at random completely, and not at random [27]. Missing value imputation brings great convenience for analyzing incomplete data. There are two commonly used technologies in terms of missing value imputation. One is using mean, median, or regression model based on statistical techniques, and the other is based on machine learning methods such as K-nearest neighbor and neural networks. While approaches based on machine learning perform better, they also tend to require a higher computational cost. The dataset in our research appears to be a high proportion of missing values, with almost all cases being incomplete (only 303 of 91713 cases are completely observed). There are 95 features have a missing percentage of at least 20%, and this means half of the features that have a missing percentage of below 20%. The imputation work consists of two steps. First, remove features that have the missing percentage exceeding 20%. There are two types of features in our dataset, continuous data such as records of body temperature, and category data such as whether the patient had an acute renal failure during the first 24 hours of their unit stay. Generates multivariate imputations by chained equation (MICE) algorithm implements multiple imputations using the fully conditional specification, which can impute the mixture features of categorical and continuous. The function “mice” within the R package MICE [27] is used to implement the multivariate imputations for missing values, and the function “with” was used to compare the complete data.

The imbalanced structure of the dataset makes mortality prediction challenging. Handle problem of imbalance is a primary step for classification. There are two commonly used methods for handling the problem of imbalance. One is based on the random oversampling (undersampling) technique by increasing (decreasing) the number of minority samples to improve the effect of the algorithm [19]. The other one is to improve the classification performance of the algorithm itself. Recently, results in terms of class imbalance are proposed by researchers, such as the algorithm based on the clustering idea and a method combined with tree-based models. Here, the oversampling method is used to get a balanced dataset.

The article "Mortality prediction in ICU Using a Stacked Ensemble Model" was published in 2022. Journal: Comput Math Methods Med.

### 3.3. Feature Selection

High-dimensional data exists in various fields, such as finance, biotechnology, and clinical research. Conventional approaches reach their limited performance due to the characteristic of high dimensionality. This section deals with high-dimensional features from two perspectives. One selects subset features using correlation analysis, and the other maps high-dimensional features into a lower space through linear transformation [22].

#### 3.3.1. The Subset Selection Method

The subset selection method is to retain the features with high correlation by performing a series of feature filtering and correlation selection on the original data. The detailed process is as follows: The chi-square test [13] is widely used to assess the correlation between two categorical variables. Defined the chi-square test statistics

(2) $$\begin{array}{c} \chi^{2}=\overset{n}{\underset{i=1}{\sum }}\frac{{\left(A_{i}-T_{i}\right)}^{2}}{T_{i}}. \end{array}$$

The *A*_*i*_ indicates the observed number, and the *T*_*i*_ indicates the theoretical number. The high value of statistics means a strong correlation between two features. The categorical features within the subset are selected through the *χ*^2^ test. The Pearson correlation coefficient is a widely used indicator that can describe the degree of linear correlation between two variables. The high value indicates the strong correlation between two variables. The subset features are selected according to some given threshold value based on the correlation matrix.

#### 3.3.2. The Transformation Method

From the perspective of dimensionality reduction, the method used for feature selection is the transformation technology which maps the high-dimensional space to the low-dimensional space. The transformation includes linear and nonlinear, both of which aim to represent most of the information in the original feature with fewer features and remove the noise information. Techniques based on nonlinear transformations, such as t-distribution random neighborhood embedding (T-SNE) [22]. Principal component analysis (PCA) is a commonly used unsupervised technique based on linear transformation, in which new features are generated.

The widely used statistical technique is still principal component analysis (PCA), although improved versions based on PCA have been proposed in recent years. Due to the availability, conventional PCA techniques are used for dimension reduction in the following research.

The article "Mortality prediction in ICU Using a Stacked Ensemble Model" was published in 2022. Journal: Comput Math Methods Med.

### 3.4. The Framework of SEM

Ensemble learning is a commonly used technology, which combines several base models into an integrated model for the improvement of learning efficiency. Commonly used ensemble techniques include bagging, boosting, and stacking [28]. Random forest [11] is a typical ensemble model based on bagging, in which the final result is obtained by voting on the different results obtained by the decision tree on random subsets of training data. Unlike the bagging method, the stacked model integrates several heterogeneous algorithms into a single model using stacking technology, which focuses on the good ones and discredits the bad ones [28]. Compared with other ensemble techniques, the stacking method is more flexible in handling different types of base models and accessible to implement due to its hierarchical structure.  Figure 1 shows the framework of the stacked ensemble model. The stacking integration process is mainly accomplished in two steps. First, predictions on the training set are obtained using the k-fold cross-validation for each base model to prevent overfitting. Taking the predictions generated by the first step as the new training data to establish the second layer, logistic regression is generally employed to get the final prediction.

The feature AHDP and AIDP represent two types of predicted probability for hospital and ICU deaths based on the APACHE 3 score and other covariates. Fortunately, the statistical test shows that both of them have significant effect on ICU mortality. It is essential to use the two features to improve model prediction. A natural idea is to integrate an ensemble model by using the corresponding probabilities of these two features. To improve the interpretability of the proposed SEM, LR, NB, RF, and XGB are employed to train weak classifiers, denoted as ALR, ANB, ARF, and AXGB. Finally, the proposed SEM model was constructed by integrating the base learner LR, NB, RF, XGB, and AXGB. For the future work, to improve the model performance, deep learning techniques such as CNN could be considered as the basic learner for building ensemble models. The framework of APACHE-based model is given in Figure 2 and the algorithms in detail are given as follows.

## 4. Empirical Studies

This section presents the experimental and analytical results of the proposed model. Several R packages [29] are used to execute the experiment. In terms of the data preprocessing, caret and MICE [27] packages are used to achieve all experiments. LR is performed using the glmnet [30] package. NB is performed using the klaR [31] package and the random forest [11] package is used to execute the RF algorithm. The packages XGBoost [32] and SHAPforxgboost [33] are used to perform the XGB algorithm and SHAP analysis, respectively. There is no existing package to handle the stack algorithm. The framework in H2O [34] package is used to model the proposed stacked algorithm. Finally, model evaluation is performed using the package pROC [35].

The article "Mortality prediction in ICU Using a Stacked Ensemble Model" was published in 2022. Journal: Comput Math Methods Med.

### 4.1. Description Analysis

Clinical practice shows that age is an essential clinical indicator in ICU intensive care. The same diagnostic treatment programs or medical facilities have different effects on different age groups. As can be seen from Table 3, the mortality rate increases with age score.

There are two kinds of conventional approaches to deal with high-dimensional features. One is feature selection, which filters features with low relevance by retaining features with high relevance. The other is the dimensionality reduction technique, which replaces the original features with lower dimensionality by transforming the feature structure. To enhance the model performance, two feature sets are obtained based on the original feature sets, labeled as SetS and SetT. The detail information in terms of feature set are given in Table 4.

### 4.2. Model Evaluation

Two datasets are generated based on the feature set SetS and SetT. The experiments are executed on datasets, in which each dataset is divided into training data and test data using 70/30 split, and 5-fold cross-validation is performed on the training data. To evaluate the model performance, several evaluation indexes are used, such as F-score, AUC, recall, and confusion matrix [36]. The confusion matrix is composed of true positive (TP), true negative (TN), false positive (FP), and false negative (FN). The evaluation indicators based on the confusion matrix are shown in Table 5.

In [7], APACHE 4, APACHE 4, and SAPS scores are used to model mortality in emergency departments, and the results show that APACHE 4 outperformed the other two scoring systems in terms of classification. APACHE 4 is employed to model mortality in ICU, and the results show that the APACHE 4 outperformed other comparable methods [7, 37]. The feature AHDP is a probabilistic prediction of in-hospital mortality for the patient, which uses the APACHE III score and other covariates. The feature AIDH indicates the probabilistic prediction of ICU mortality for the patient which utilizes the APACHE III score and other covariates. Fortunately, both of these indicators are given as predictive probabilities, which we can naturally assume to be a type of classifier trained from the other features.

The article "Mortality prediction in ICU Using a Stacked Ensemble Model" was published in 2022. Journal: Comput Math Methods Med.

As shown in Table 6, AHDP and AIDP are used to establish the models, such as ALR, ANB, ARF, and AXGB. LR achieves poor performance due to the parallel relationship between the two features, which does not have a strong linear correlation. Compared with the conventional statistical methods, machine learning algorithms perform better because they can handle data with complex structures well, among which the AXGB model gives an AUC value of 0.868. The results ensure the effectiveness of the proposed integration model. The details in terms of the corresponding results are given in the following table.

The ensemble model takes LR, NB, RF, XGB, and AXGB as the base learner, in which AXGB is a weak learner based on the features AHDP and AIDP. Here, we choose the model AXGB as the AL in Algorithm 1 due to the model AXGB achieves the best performance compared to other models learned from AHDP and AIDP. The essence of the proposed integration model SEM is a hierarchical model with three layers. The crucial step is that the predicted values based on the 5-fold cross-validation in the first layer are used as the training data of the next layer model. It should be noted here that to maintain the unity of the integration model framework, for the base model AXGB, we directly treat its prediction results as the 5-fold cross-validation results obtained on the same original training set. LR, NB, RF, XGB, and the proposed stacked ensemble model (SEM) are used for modeling the prediction of mortality rate based on the subset feature SetS and the transformed SetT, respectively. The evaluation statistics precision, recall, F-scores, and AUC were calculated to evaluate the performance of each model.

Table 7 shows the performance of the proposed model SEM on several evaluation indicators. In order to improve the performance of prediction, the proposed ensemble model is performed on two types of feature subsets, respectively. The SEM model based on the SetS (AUC: 0.879) outperformed model based on the SetT (AUC: 0.860). Comparison results are given in Figure 3(b). In Figure 3(a), under the three model building frameworks, the proposed SEM achieves the highest AUC value of 0.879, outperforming the model without integrating the APACHE results. The above analysis results are only for the existing dataset. The performances of the model are expected to improve based on the emergence of continuously innovative methods. Improvements in data preprocessing and advanced methods of feature extraction are good ways to improve prediction. In clinical practice, mortality is influenced by more factors, and the results of the analysis based on this dataset have a particular referential value for understanding mortality in ICU.

The article "Mortality prediction in ICU Using a Stacked Ensemble Model" was published in 2022. Journal: Comput Math Methods Med.

### 4.3. Feature Importance Analysis

The importance of features is characterized by their impact on response variables. Generally speaking, the greater the impact on the outcome feature, the more important the features are. In Figure 4, the *x*-axis denotes the Shapley value, and the *y*-axis represents the features that are sorted in decreasing order of importance. Each row in the figure represents a feature, and the points in each row represent samples. The darker the color, the higher the Shapley value of the feature. As shown in Figure 4(a), AHDP and AIDP are the two most important features for modeling mortality rates. In Figure 4(b), the same analysis is performed using the features without AHDP and AIDP. Age plays a crucial role in modeling ICU mortality prediction. In the former analysis, it was obtained that the features AHDP and AIDP has a strong correlation with the mortality rate. Combined with SHAP analysis, it is may be a good strategy to construct the classifier based on the feature AHDP and AIDP. In Section 4.2, the proposed model SEM and model evaluation have confirmed the feasibility of this strategy.

### 4.4. SHAP Dependency Analysis

SHAP importance analysis explains which features contributed most to the mortality rate. In practice, risk at the same age may continuously change with other indicators. It is meaningful to determine the “threshold” at which the risk to the patient suddenly changes. SHAP dependency analysis is employed to explain the relationship between the value of the feature and the corresponding Shapley value.

Figure 5 consists of 6 subfigures. In each subfigure, the *x*-axis denotes feature values, the *y*-axis denotes the corresponding Shapley values, and the color denotes the interactive effect produced by the second feature. It can be seen from Figure 5(a), that the correlation coefficient 0.9 means that feature age had a strong relationship with its Shapley value, which means the Shapley value increased with age. The aged patients in the same conditions had a higher risk of mortality. In Figure 5(c), Shapley value gets larger with the value of feature d1_bun_min increase, after the peak value d1_bun_min =30 mmol/L, the Shapley values does not increase. In Figure 5(d), for the feature gcs_motor_apache, the Shapley contribution score decreases as the value of gcs_motor_apache take. That is because the lower score indicates the severity condition for patients. In summary, for continuous features, the risk of mortality has significantly changed in the following values: d1_bun_min>10 mmol/L, d1_heartrate_min <75 min, and d1_spo2_min<90%. For the category features, ap3diag<480 and gcs_motor_apache<4. Due to the complexity of disease control and individual differences, the efficiency that patients receive may vary from each other.

The article "Mortality prediction in ICU Using a Stacked Ensemble Model" was published in 2022. Journal: Comput Math Methods Med.

## 5. Conclusion and Discussion

With the development of science and technology, intelligent diagnosis has attracted significant attention. Combining medical experience and scientific technology to improve the efficiency of diagnosis will benefit both medical workers and patients. The research proposes a novel stacked ensemble model that attempts to combine the conventional clinical severity scoring methods with machine learning techniques to improve mortality prediction in ICU. The proposed ensemble model SEM achieves good performance compared to LR, NB, RF, and XGB. The performance on the selected subset SetS gives an AUC of 0.879, while the transformed subset SetT gives 0.860. Compared to the model without integrating the APACHE 4 prediction results, the proposed model gives a higher AUC. Furthermore, SHAP analysis is employed to interpret the contribution of features and their significance.

The performance and stability of the model are affected by various factors, such as data preprocessing, feature selection, and model structure. In the future work, the model could be constructed from the perspective of feature selection to explore the interpretation and interactivity between features and outcomes. In terms of method, taking the existing severity scoring results as prior information, combined with the machine learning algorithms to explore the mixture method may be an alternative strategy. [10] proposed a machine learning model based on the SOFA score for the prediction of mortality in critically ill patients. [38] developed a two-step Bayesian approach to optimize clinical decisions on timing, and the result shows that the proposed model are clinically useful to improve the survival of patients. The model of the research can be extended to other severity scoring systems, such as SOFA, GCS, and CT. It is expected that innovative combination strategies can be proposed to boost the performance of the model.

## Figures and Tables

**Figure 1:** The framework of stacked ensemble model. In Figure 1(a), five groups of predictions based on 5-fold cross validation are used as the new training set. In Figure 1(b), logistic regression is used for modeling the new training set.

**Figure 2:** The framework of features and approaches in the experiment. The blue rectangle icons represent feature sets, and the orange ellipse icons represent approaches.

**Figure 3:** Model performance on test data. (a) Compared with three models, the proposed SEM is superior to others, which has the AUC of 0.879 and 95% CI (0.842,0.883). (b) The performance of SEM based on SetS achieves better prediction.

The article "Mortality prediction in ICU Using a Stacked Ensemble Model" was published in 2022. Journal: Comput Math Methods Med.

**Figure 4:** The rank of feature importance based on the SHAP contribution values. Figure 4 shows the top 10 important features based on the Shapely contribution values. The feature AHDP and AIDP have a strong relationship with the mortality rate.

**Figure 5:** SHAP interaction analysis plots of the selected features. Abbreviation: ap3diag: apache_3j_diagnosis. (a) The interaction analysis for age and its corresponding SHAP value. (b) The interaction analysis for ap3diag and its corresponding SHAP value. (c) The interaction analysis for d1_bun_min and its corresponding SHAP value. (d) The interaction analysis for gcs_motor_apache and its corresponding SHAP value. (e) The interaction analysis for d1_heartrate_min and its corresponding SHAP value. (f) The interaction analysis for d1_spo2_min and its corresponding SHAP value.

**Algorithm 1:** APACHE score-based model using stacked ensemble technique.

**Table 1:** Example of related literature and technical comparison.

References	Technique	Characteristics
[1]	Weight decay RF, integrate the missing value analysis and likelihood ratio test.	Based on sparse data, robust calibration for large-scale dataset.
[7]	APACHE IV scoring system method	Weak calibration for new data records.
[10]	SOFA-based ML, (XGBoost, RF, SVM, and LR)	Comparison with four different ML approaches, incorporating the time information.
[12]	LR and ensemble techniques.	Poor performance for the nonlinear relationship
[13]	XGBoost	Improved accuracy and applicability; promising performance for nonlinear relationship; SHAP analysis for interpreting the model.
[16]	Deep learning(rnn)	Learn complex interactions from the data; reduced explainability for the model.

**Table 2:** Examples of features in different types and the corresponding description of missing values.

Class	Name	Unit	Missing percentage (%)
Demographics	Age	Years	4.6
	BMI	kilograms/metres^2^	3.7
	PILD	1	0
	⋯	⋯	⋯
Vital signs	d1_heartrate_max	Beats per minute	3
	d1_spo2_max	Percentage	0.4
	d1_temp_max	Degrees Celsius	23.7
	⋯	⋯	⋯
Laboratory features	h1_bun_min	g/L	11.5
	d1_albumin_min	g/L	91.4
	d1_glucose_max	mmol/L	57.4
	⋯	⋯	⋯
APACHE covariates	gcs_motor_apache	None	2.1
	heart_rate_apache	None	1
	⋯	⋯	⋯
APACHE comorbidity	Leukemia	None	0.8
	sodium_apache	mmol/L	0.8
	Aid	None	0.8
	diabetes_mellitus	None	0.8
	Immunosuppression	None	0.8
	⋯	⋯	⋯
APACHE prediction	AHDP	None	8.7
	AIDP	None	8.7

Abbreviation: PILD: pre_icu_los_days; AHDP: apache_4a_hospital_death_prob; AIDP: apache_4a_icu_death_prob.

The article "Mortality prediction in ICU Using a Stacked Ensemble Model" was published in 2022. Journal: Comput Math Methods Med.

**Table 3:** Mortality rate at different age score risk levels.

Age segmentation	<44	45-54	55-64	65-74	>75
Scores	0	2	3	5	6
Mortality rate	0.049	0.056	0.073	0.092	0.128

**Table 4:** Feature selection results based on two approaches.

Feature sets	Approaches	Numbers
SetS	Correlation filtering method	80
SetT	PCA	54

**Table 5:** Calculation formulas for evaluation indicators.

Indicators	Formulas
Precision	$\frac{\text{TP}}{\text{TP}+\text{FP}}$
Recall	$\frac{\text{TP}}{\text{TP}+\text{FN}}$
F-scores	$\frac{2\text{TP}}{2\text{TP}+\text{FN}+\text{FN}}$

**Table 6:** Performance of several methods based on feature AHDP and AIDP.

Feature set	Model	Precision	Recall	AUC	F-scores
AHDP, AIDP	ALR	0.916	0.633	0.623	0.564
	ANB	0.923	0.635	0.746	0.632
	ARF	0.917	0.714	0.646	0.712
	AXGB	0.919	0.823	0.868	0.823

**Table 7:** Performance of different methods based on two feature sets.

Feature set	Model	Precision	Recall	AUC	F-scores
SetS	LR	0.914	0.633	0.632	0.564
	NB	0.745	0.635	0.745	0.632
	RF	0.677	0.714	0.677	0.712
	XGB	0.924	0.823	0.862	0.823
	SEM	0.924	0.831	0.879	0.824
SetT	LR	0.623	0.654	0.648	0.634
	NB	0.612	0.65	0.636	0.651
	RF	0.734	0.735	0.721	0.712
	XGB	0.812	0.856	0.823	0.823
	SEM	0.816	0.862	0.860	0.845

## Data Availability

The source code in the method is available from the first author upon request. WiDS dataset is available at doi:10.13026/vc0e-th79.
